RETRACTED

# Skin barrier dysfunction measured by transepidermal water loss at 2 days and 2 months predates and predicts atopic dermatitis at 1 year

**DOI:** 10.1016/j.jaci.2014.12.013

**Published:** 2015-04

**Authors:** Maeve Kelleher, Audrey Dunn-Galvin, Jonathan O'B. Hourihane, Deirdre Murray, Linda E. Campbell, W.H. Irwin McLean, Alan D. Irvine

**Affiliations:** a Paediatrics and Child Health, University College Cork, Cork, Ireland; b National Children's Research Centre, Dublin, Ireland; c Dermatology and Genetic Medicine, University of Dundee, Dundee, United Kingdom; d Paediatric Dermatology, Our Lady's Children's Hospital, Dublin, Ireland; e Clinical Medicine, Trinity College Dublin, Dublin, Ireland

**Keywords:** Infant, skin barrier, TEWL, atopic dermatitis, filaggrin, predictor, biomarker, AD, Atopic dermatitis, AUC, Area under the ROC curve, BASELINE, Babies After Scope: Evaluating the Longitudinal Impact Using Neurological and Nutritional Endpoints, *FLG*, Filaggrin gene, LR, Logistic regression, OR, Odds ratio, ROC, Receiver operating characteristic, SCOPE, Screening for Pregnancy Endpoints, TEWL, Transepidermal water loss, ΔTEWL, Change in TEWL measurement between one timepoint and another

## Abstract

**Background:**

Loss-of-function mutations in the skin barrier protein filaggrin (*FLG*) are a major risk for atopic dermatitis (AD). The pathogenic sequence of disturbances in skin barrier function before or during the early development of AD is not fully understood. A more detailed understanding of these events is needed to develop a clearer picture of disease pathogenesis. A robust, noninvasive test to identify babies at high risk of AD would be important in planning early intervention and/or prevention studies.

**Objectives:**

To ascertain whether a noninvasive measurement of skin barrier function at day 2 after birth and at 2 months predicts the development of AD at 1 year. Furthermore, to determine whether increases in transepidermal water loss (TEWL) predate the development of clinical AD.

**Methods:**

A total of 1903 infants were enrolled in the Cork Babies After Scope: Evaluating the Longitudinal Impact Using Neurological and Nutritional Endpoints Birth Cohort study from July 2009 to October 2011. Measurements of TEWL were made at birth (day 2) and at 2 and 6 months. The presence of AD was ascertained at 6 and 12 months, and disease severity was assessed by using the SCORing Atopic Dermatitis clinical tool at 6 months and by using both the SCORing Atopic Dermatitis clinical tool and Nottingham Severity Score at 12 months. A total of 1300 infants were genotyped for *FLG* mutations.

**Results:**

At 6 months, 18.7% of the children had AD, and at 12 months, 15.53%. In a logistic regression model, day 2 upper quartile TEWL measurement was significantly predictive of AD at 12 months (area under the receiver operating characteristic curve, 0.81; *P* < .05). Lowest quartile day 2 TEWL was protective against AD at 12 months. An upper quartile 2 month TEWL was also strongly predictive of AD at 12 months (area under the receiver operating characteristic curve, 0.84; *P* < .05). At both ages, this effect was independent of parental atopy, *FLG* status, or report of an itchy flexural rash at 2 months. Associations were increased when parental atopy status or child *FLG* mutation status was added into the linear regression model.

RETRACTED

**Conclusions:**

Impairment of skin barrier function at birth and at 2 months precedes clinical AD. In addition to providing important mechanistic insights into disease pathogenesis, these findings have implications for the optimal timing of interventions for the prevention of AD.

Atopic diseases include atopic dermatitis (AD), food allergy, allergic rhinitis, and asthma.^1^ The prevalence of these diseases has increased in recent decades, causing considerable morbidity in childhood.^2-5^ The putative “Atopic March” refers to the typical sequence of clinical manifestation of atopic disease, usually initiated by AD from early infancy.^6,7^

Parental atopy is an independent risk factor for the development of atopic disease.^8^ The genetic mechanisms and inheritance pattern of atopic diseases are not fully elucidated, but recent candidate gene studies and genomewide association studies have yielded some insights.^9^ The most widely replicated and most significant gene to influence AD is filaggrin (*FLG*).^10^ Filaggrin is a filament-binding protein in the stratum corneum.^11^ *FLG* loss-of-function mutations occur in 10% of Europeans, imparting an increased risk of AD, food allergy, and asthma.^12,13^ The overall increase in the risk of AD conferred by a single *FLG* loss-of-function mutation is approximately 3.3,^14^ with a significant additional and independent effect conferred by intragenic copy number variations in *FLG*.^15^ Importantly, *FLG* mutations increase the risk of developing asthma only in the presence of AD.^13^

The stratum corneum contributes greatly to skin barrier function. Transepidermal water loss (TEWL) is a noninvasive *in vivo* measurement of water loss across the stratum corneum.^16^ It is raised in subjects with AD.^13^ This is seen at both lesional and nonlesional skin sites.^17,18^ Recent studies of high-risk atopic individuals showed that a raised TEWL may precede the clinical manifestation of AD in those at high risk of atopy.^19^ A defect in skin barrier function may facilitate allergen entry and immune priming.^20^ Further evidence for this theory has been gained from murine studies in which systemic allergic reactions to peanut can be induced by epicutaneous sensitization across a disrupted stratum corneum.^21^ Such a defect has been proposed as a risk factor and a route of sensitization for the development of peanut allergy.^22^ With regard to aeroallergens, in a cross-sectional study of children, an increased TEWL is associated with increased sensitization to aeroallergens.^23^

RETRACTED

Currently, no primary preventative therapies have been established for AD. Given the role of filaggrin, pilot studies have focused on therapies or interventions that may enhance the infant skin barrier.^24^ Very recently 2 studies have shown that application of moisturizer in the neonatal period holds promise for the prevention of AD.^25,26^ To date though, apart from family history, there is no way of accurately identifying which children may be at the greatest risk of AD and who might therefore benefit most from intervention. In this study, we sought to determine whether a rapid and noninvasive test such as TEWL, measured at day 2 and month 2, could predict the development of AD at 12 months. Given the well-established role of *FLG* mutations, we included genetic status in our predictive model and we also included parental atopy.

## Methods

### Study subjects

The Cork Babies After Scope: Evaluating the Longitudinal Impact Using Neurological and Nutritional Endpoints (BASELINE) Birth Cohort study is the first birth cohort study in Ireland.^27^ It was developed as the pediatric follow on from the Cork Centre for the Screening for Pregnancy Endpoints (SCOPE) study, a multicenter international study evaluating diseases of pregnancy in primigravidous women.^28^ The Cork BASELINE Birth Cohort study recruited from August 2009 through to October 2011. Infants recruited from July 2009 had skin barrier assessment at birth and throughout early life; these 1903 infants are included in this study.

A total of 1303 infants were recruited antenatally (stream1). These women were subject to the inclusion criteria of the SCOPE study, namely, first-time, low-risk mothers with singleton pregnancies delivered at or near term. Consent for recruitment was sought at 20 weeks of gestation and confirmed at birth of the live baby. Cord blood samples were taken at birth and stored for future use. A second recruitment stream began in July 2010 that recruited mothers and babies on the postnatal ward (stream2). A total of 600 infants were recruited postnatally. These mothers were enrolled independently of the SCOPE study. The sole inclusion criterion in stream 2 was a healthy term infant on the postnatal ward. Stream 1 and stream 2 infants were assessed and followed up in an identical fashion at birth and thereafter clinic visits at 2, 6, and 12 months.

RETRACTED

All infants had assessment at birth, 2 months, 6 months, and 12 months involving parental questionnaires and physical assessment. Parental questionnaires at 2, 6, and 12 months contained specific screening questions for AD. Experienced health care personnel diagnosed AD at 6 and 12 months in accordance with the UK Working Party diagnostic criteria.^29-31^ If AD was present, severity was assessed at these timepoints using the SCORing Atopic Dermatitis (SCORAD) clinical tool.^32,33^ At 12 months, the Nottingham Severity Score was also recorded to assess the severity of AD.^34^

### TEWL measurements

TEWL measurements were carried out using a widely validated open chamber system (Tewameter TM 300; Courage+Khazaka Electronic, Cologne, Germany). For newborns, TEWL was taken in the Cork University Maternity Hospital. The subject's arm was acclimated before measurement by exposing the arm in a nonenvironmentally controlled room for 10 minutes. This was typically done in the cot beside the mother's bed while an interview with the mother or parents was carried out. The infant was then brought to a windowless room in which both temperature and humidity were maintained constant by an air conditioning system. Temperature was set between 20°C and 25°C. Humidity was monitored by a manometer in the room and was maintained between 30% and 45%. TEWL was taken on the lower volar surface of the forearm by applying a probe to the exposed volar skin for approximately 15 seconds until the measurement was recorded. Three readings were taken, and the mean of the 3 readings was recorded. For TEWL readings at other timepoints, the same procedure was carried out at 2 months and 6 months in an environmentally controlled room in the Health Research Board Discovery Centre, the clinical research facility for children at Cork University Hospital. The parents were advised not to apply emollients to the infant's skin for 12 hours before the reading was taken.

### Statistical analysis

A series of logistic regression (LR) models was used to estimate the factors at (1) 2 days and (2) 2 months that influence the diagnosis of AD at 12 months. The dependent variable that measures diagnosis at 12 months is AD “Yes” and is equal to 1, with AD “No” = 0. To examine the influence of each variable, with and without the presence of other significant predictors, we carried out both univariable and multivariable analyses. With regard to the latter, 3 models were produced. Model 1 included parental atopy, *FLG* mutation status, and presence of an itchy rash at 2 months as independent variables. Model 2 included parental atopy and TEWL test reading scores at 25th, 50th, and 75th percentiles (7.0, 9.4, and 12.3, respectively) as independent variables, but did not include *FLG* mutation status. This was done to determine the unique influence of TEWL, without the contribution of *FLG* mutations. Model 3 included all independent variables: parental atopy, TEWL test reading scores, and *FLG* mutation status. All models controlled for the variables “use of emollient before test reading,” “presence of an itchy rash,” “infant sex,” and “infant birthweight.” Receiver operating characteristic (ROC) curve output, which plots the true positives (sensitivity) vs false positives (1 − specificity), was then evaluated to compare the ability of the 3 models to produce a prognosis with high accuracy. Our rationale for variable selection was to include those predictors necessary for face validity but only if they were significant at a .05 level in the univariable analysis or if they altered the coefficient of the main variable by more than 10% in cases in which the main association was significant.^35,36^

RETRACTED

## Results

A total of 1903 infants were enrolled onto the study. The demographic details of the population studied are presented in Table I.

### Filaggrin mutation typing

Stream 1 infants had cord blood samples taken at birth. Infants without cord blood samples had Oragene saliva samples taken. Those infants still enrolled in the study at 2 years had EDTA blood samples taken. *FLG* genotyping was carried out in 1300 infants with available DNA. The cumulative *FLG* mutation rate was 10.46% (136 of 1300). Four infants were homozygous for *FLG* mutation, with the remainder heterozygous for *FLG* mutation (Table II).

### TEWL through early infancy

TEWL was taken in the early newborn period in 1691 of 1903 (88.86%) infants of the cohort. The mean TEWL for newborns was 7.32 ± 3.33 g_water_/m^2^/h. Using univariable analysis, we found that there was no significant association between TEWL measurements at birth and sex, gestation, or postnatal age at measurement or recruitment stream 1 or 2 (data not shown). A total of 1614 of 1638 (98.5%) infants who attended the 2-month appointment had TEWL measured (98.5%). Mean 2-month TEWL was 10.97 ± 7.98 g_water_/m^2^/h. A total of 1516 of 1537 (98.6%) infants who attended the 6-month appointment had TEWL measured. Mean 6-month TEWL was 10.71 ± 7.10 g_water_/m^2^/h. TEWL measurements by quartiles are presented in Table III.

### Clinical diagnosis of AD

AD was screened for at 6- and 12-month appointments. This diagnosis of AD was made according to the UK Working Party diagnostic criteria. At 6 months, 18.7% (299 of 1597) of the infants screened were diagnosed with AD. A total of 287 had a SCORAD completed, with a mean SCORAD score of 21.54 ± 16.29 (range, 0-88). At 12 months, 15.53% (232 of 1494) of the infants screened were diagnosed with AD. The mean SCORAD score at 12 months in affected children was 18.56 ± 14.92 (range, 0-77).

RETRACTED

### LR analysis: Factors influencing the development of AD at 1 year

Our primary outcome was the presence of AD at 1 year. We developed a model that explored the relative contributions of *FLG* mutation status, parental atopy, presence of an itchy rash at 2 months, TEWL at day 2 and month 2, and ΔTEWL (day 2 to month 2 and day 2 to month 6) on AD at 1 year (Table IV). *FLG* mutation status was not associated with an elevated TEWL at birth. However, it was associated with an elevated TEWL at 2 and 6 months and with elevated ΔTEWL day 2 to 2 months and ΔTEWL day 2 to 6 months. Notably, *FLG* mutation carriers did not have elevated ΔTEWL 2 months to 6 months, implying that the major changes in skin barrier function in those who develop AD by 12 months start in the first 2 months of life. In our univariable modeling, the odds ratio (OR) for AD at 12 months conferred by both parents being atopic was 2.5 compared with an OR of 3.1 for an upper quartile TEWL at 2 months (see Table E1 in this article's Online Repository at www.jacionline.org). LR models were then used to examine the factors at birth and at 2 months that influence a diagnosis of AD at 12 months. We used 3 separate models to explore the relative contribution of parental atopy, *FLG* mutation status, and TEWL (at day 2 and at 2 months) toward the development of AD at 12 months. All models controlled for the variables use of emollient before test reading, presence of an itchy rash, infant sex, and infant birthweight. These covariates were not significant in any of the 3 multivariable models.

### LR modeling of AD risk at 12 months including day 2 TEWL

The LR model incorporating day 2 TEWL is summarized in Table V. In our first model, we included parental atopy and *FLG* mutation status as independent variables and excluded day 2 TEWL. Parental atopy and *FLG* mutation status significantly increase the likelihood of a positive diagnosis of AD at 12 months by 13.7 and 8.6 times, respectively, compared with infants without *FLG* mutation and without an atopic parent. The ROC, which plots the true positives (sensitivity) vs false positives (1 −specificity), is 0.8 for this model. Our second model includes day 2 TEWL test reading scores at 25th, 50th, and 75th percentiles as independent variables. We did not include *FLG* mutation status in this second model. The area under the ROC curve (AUC) remains at 0.8 for this model. Infants with a TEWL reading of 9.0 or above are 7.1 times more likely to be diagnosed with AD at 1 year than are infants with a reading below this point, controlling for all other variables in the model. This suggests that day 2 TEWL can be used as a sole indicator of likelihood of AD at 12 months. Our third model includes all independent variables, including both TEWL and *FLG* status.

RETRACTED

### LR modeling of AD risk at 12 months including TEWL at 2 months

We repeated the LR approach for month 2 TEWL values, summarized in Table VI. Again, we used 3 models. In the first model, we included parental atopy and *FLG* mutation status as independent variables but did not include TEWL. Parental atopy and *FLG* mutation carriage significantly increase the likelihood of a positive AD diagnosis at 12 months by 2.7 and 3.0 times, respectively, compared with infants without an *FLG* mutation and without an atopic parent. The ROC is 0.66 for this model. In the second model, we included the month 2 TEWL test reading scores at 25th, 50th, and 75th percentiles (7.0, 9.4, and 12.3 g_water_/m^2^/h, respectively) as independent variables. We did not include *FLG* mutation status in this second model, as explained above. The AUC improved from 0.66 to 0.82 in this model. Infants with a TEWL reading of 12.3 or above were 5.6 times more likely to be diagnosed with AD at 12 months than were infants with a reading below this point, controlling for all other variables in the model. Model 3 included all independent variables. In a pattern similar to that found at 2 days, the AUC improved slightly to 0.84, although here again it is important to note that model 2 demonstrates that *FLG* status need not be measured to produce a prognosis with high accuracy. We modeled these in a traditional stepwise LR analysis. The significant finding was that after controlling for all other possible influencing factors, month 2 TEWL was the strongest independent predictor of AD at 12 months.

## Discussion

This study involves a large, unselected birth cohort study and is the first study of this scale to assess skin barrier function in the newborn period and early infancy. We have shown that changes in skin barrier predate clinical AD with a signal for barrier impairment detected in asymptomatic infants at day 2 and more markedly at 2 months. In our univariable modeling, the OR for AD at 12 months conferred by both parents being atopic was 2.5 compared with an OR of 3.1 for an upper quartile TEWL at 2 months (see Table E1), showing the additional value of an TEWL reading at this stage. These changes are seen in both high-risk and low-risk infants and, crucially, are independent of *FLG* status. Although in our multivariable analysis the AUC improves slightly to 0.83 when all available variables are included, importantly our second model (which excludes *FLG* genotyping) demonstrates that *FLG* status need not be measured to produce an accurate 12-month AD prognosis for babies with upper quartile day 2 TEWL readings.

RETRACTED

Some children will develop AD before 6 months. In our study, we did not formally diagnose AD at 2 months but all parents were asked about the presence of itchy rash on face or skin folds. These infants were designated as “itchy rash,” seen in 8% of all cases at 2 months. There are no widely recognized diagnostic criteria for AD at this age; however, we controlled for an itchy red rash at the 2-month visit in our model. AD was screened for in all participants at 6 and 12 months and formally diagnosed using the UK Working Party Criteria. When compared with other studies in the field, our study shows the earliest timepoint for a signal for impaired TEWL in asymptomatic infants: at day 2. A further, stronger signal is seen at 2 months.

Previous studies, of smaller scale have shown a relationship between *FLG* mutation status and TEWL.^19^ However, our study is much larger, by several orders of magnitude, and is not selected for high risk of atopy. In our study, 30% of *FLG* mutation carriers developed AD by age 12 months and 70% did not, consistent with large previous studies. At birth, there was no difference in mean TEWL reading between *FLG* mutation and *FLG* wild-type groups (7.33 ± 3.62 g_water_/m^2^/h vs 7.3 ± 3.38 g_water_/m^2^/h). However, by 2 months, *FLG* mutation carrying infants have a significantly higher mean TEWL than do *FLG* wild-type infants. This change persisted at 6 months.

Selecting out children in the upper quartile regardless of *FLG* status allows for a noninvasive, discriminating, and targeted means of prediction of AD in the first days of life, allowing for possible preventive measures to be put in place. Conversely, selecting out infants in the lower quartile of TEWL, which has a protective effect in relation to AD at 12 months, could be an important piece of positive information for their families and would reduce the “number needed to treat” in an intervention study of potential protective interventions. Detection of an increased TEWL as early as day 2 or at 2 months, before developing clinical features of AD, is a novel and unique finding in a general pediatric population. Accurate identification of individuals at high risk for AD, using family history in combination with a noninvasive measurement, with the optional addition of *FLG* mutation status has great potential for intervention studies. Stratified interventions could be made on the basis of these 2 or 3 variables. Pilot studies for the primary prevention of AD by use of liberal emollients have shown the potential of this approach.^24^ We believe that the novel findings in this study will facilitate and inform stratification of future intervention studies.

RETRACTED

A lowest quartile TEWL at birth is protective against AD. A highest quartile TEWL at 2 days and at 2 months is strongly associated with increased prevalence of AD at 12 months. These changes predate the development of clinically apparent AD. The mechanistic implications of these observations are that abnormalities in the skin barrier predate symptomatic or clinically detectable AD. These changes occur very early in the postnatal environment after transition from the intrauterine aqueous environment to the xerotic postnatal environment. It is notable that this effect is not dependent on *FLG* loss-of-function mutations but is enhanced by and is interactive with these genetic factors and presumably with environmental influences encountered postnatally. TEWL measurement in early life is therefore an effective tool to detect infants at risk of AD, especially when combined in a model with parental history of atopy and/or *FLG* mutation status. The obvious next step would be to assess whether intervention studies between birth and age 2 months in those with raised TEWL at birth would be effective in maintaining the skin barrier and reducing the incidence of AD.

**Clinical implications**

A signal for the development of AD is seen at 2 days and at 2 months in asymptomatic infants. Interventions to potentially prevent AD could be targeted toward such infants.

## Figures and Tables

**Table E1:** Univariate table

Variable	OR	CIs	*P* value
TEWL birth percentiles			
25^th^ (5.0 g_water_/m^2^/h)	—		
50^th^ (7.0 g_water_/m^2^/h)	1.9	1.27-2.86	.002
75^th^ (9.0 g_water_/m^2^/h)	1.6	1.10-2.53	.03
TEWL 2-mo percentiles			
25^th^ (7.0 g_water_/m^2^/h)	—		
50^th^ (9.4 g_water_/m^2^/h)	1.4	0.95-1.95	.9
75^th^ (12.3 g_water_/m^2^/h)	3.1	2.21-4.22	.0001
Parental atopy			
None	—		
One (yes)	1.4	1.03-2.01	.03
Both (yes)	2.5	1.67-3.66	.0001
Visible rash at 2 mo (yes)	2.7	1.88-4.1	.001
*FLG* loss-of-function mutation (yes)	2.9	1.94-4.45	.0001
Use of emollient	1.1	0.6-2.4	.1
Baseline 1 vs 2	1.1	0.9-1.53	.3
Birthweight	1.01	1.0-1.2	.4
Sex	0.91	0.7-1.2	.4

**Table I:** Baseline demographic characteristics

Characteristic	Value
Total enrolled	1903
Sex: male/female (%)	50.4/49.6
Birthweight (g), mean ± SD	3489 ± 512
Gestation (d), mean ± SD	279.33 ± 10.77

RETRACTED

**Table II:** *FLG* mutation rates

*FLG* mutation	Heterozygous rate (%)	Homozygous rate (%)	Total (%)
R501X	4.0 (52 of 1300)	0.23 (3 of 1300)	4.23 (55 of 1300)
2282Del4	3.62 (47 of 1300)	0	3.6 (47 of 1300)
S3247X	1.54 (20 of 1300)	0.08 (1 of 1300)	1.62 (21 of 1300)
R2447X	1 (13 of 1300)	0	1 (13 of 1300)
*FLG* mutation (total)	10.15 (132 of 1300)	0.31 (4 of 1300)	10.46 (136 of 1300)

**Table III:** TEWL by quartile at day 2 and month 2

	Birth TEWL	% of total sample	2-mo TEWL test score value	% of total sample
Mean	7.3		10.9	
Median	7.0		9.4	
Mode	5.0		10.0	
SD	3.3		7.9	
Minimum	0.4		0.8	
Maximum	34.0		92.3	
Percentiles				
25	5.0	45	7.0	43
50	7.0	27	9.4	21
75	9.0	28	12.3	36

**Table IV:** Relationship between *FLG* status and mean TEWL values

	Mean TEWL (g_water_/m^2^/h)		*P* value
	*FLG* wild-type	*FLG* mutation	
N	1164	136	
Birth	7.3 ± 3.38	7.33 ± 3.62	.91
2 mo	10.7 ± 7.7	12.6 ± 10.1	.04
6 mo	10.42 ± 7.1	12.25 ± 6.53	.007
Δ Birth to 2 mo	3.32 ± 8.1	5.44 ± 10.66	.046
Δ Birth to 6 mo	2.93 ± 7.55	4.62 ± 7.11	.03
Δ 2 to 6 mo	0.35 ± 10.11	0.75 ± 9.95	.685

**Table V:** LR model for factors at birth influencing AD at 12 months

Predictor variable at birth	OR; CI (*P* value)		
	Model 1	Model 2	Model 3
Parental atopy			
None	—	—	—
One (yes)	10.2; 1.4-11.8 (.05)	1.7; 0.5-4.8 (.2)	11.5; 0.3-5.6 (.1)
Both (yes)	13.7; 1.0-25.4 (.05)	9.0; 4.4-20.4 (.001)	13.4; 1.2-14.0 (.1)
*FLG* loss-of-function mutation			
No	—	—	—
Yes	8.6; 1.1-24.7 (.02)	—	10.2; 1.2-18.5 (.3)
TEWL birth percentiles			
25th (5.0 g_water_/m^2^/h)	—	—	—
50th (7.0 g_water_/m^2^/h)	—	3.2; 0.9-15.0 (.07)	1.9; 0.3-17.7 (.9)
75th (9.0 g_water_/m^2^/h)	—	7.1; 1.8-12.9 (.001)	6.9; 0.6-34.3 (.1)
Adjusted for			
Use of emollient (yes)	0.8; 0.3-2.5 (.8)	0.8; 0.3-2.0 (.6)	0.7; 0.2-2.2 (.7)
Sex (male)	0.9; 0.3-4.0 (.7)	0.8; 0.3-1.9 (.6)	0.9; 0.3-2.5 (.8)
Birthweight	1.0; 0.9-1.1 (.5)	1.0; 0.9-1.1 (.5)	1.0; 0.9-1.1 (.5)
Visible itchy rash	1.3; 0.3-5.9 (.7)	2.1; 0.7-6.3 (.2)	0.7; 0.2-3.2 (.6)
Baseline 1 vs 2	2.8; 0.7-11.5 (.2)	2.3; 0.6-8.1 (.2)	3.1; 0.7-13.2 (.2)
Model χ^2^ statistic for overall model fit	18.5 (.05)	14.7 (.04)	16.3 (.05)
AUC	0.8; 0.7-0.9 (.01)	0.8; 0.7-0.9 (.01)	0.83; 0.7-0.9 (.01)

Controlling for “use of emollient before test reading,” “visible itchy rash at 2 months,” “infant sex,” and “infant birthweight.”

**Table VI:** LR model for factors at 2 months influencing AD at 12 months

Predictor variable at birth	OR; CI (*P* value)		
	Model 1	Model 2	Model 3
Parental atopy			
None	—	—	—
One (yes)	1.4; 0.4-2.7 (.6)	1.7; 0.5-4.8 (.2)	1.5; 0.3-5.6 (.1)
Both (yes)	2.7; 1.3-4.1 (.01)	9.0; 4.4-20.4 (.001)	6.5; 1.2-14.0 (.01)
*FLG* loss-of-function mutation			
No	—	—	—
Yes	3.1; 2.0-4.9 (.02)	—	2.9; 0.4-19.5 (.28)
TEWL 2-mo percentiles			
25th (7.0 g_water_/m^2^/h)	—	—	—
50th (9.4 g_water_/m^2^/h)	—	1.1; 0.3-3.8 (.9)	1.5; 0.3-4.1 (.9)
75th (12.3 g_water_/m^2^/h)	—	5.6; 1.8-12.9 (.001)	7.9; 1.7-25.0 (.01)
Adjusted for			
Use of emollient (yes)	1.1; 0.3-3.5 (.8)	1.2; 0.4-3.1 (.7)	0.5; 0.5-6.1 (.3)
Sex (male)	0.9; 0.3-2.4 (.7)	0.9; 0.3-2.1 (.6)	0.9; 0.8-1.1 (.8)
Birthweight	1.0; 0.9-1.0 (.3)	1.0; 0.9-1.0 (.4)	0.9; 0.8-1.0 (.3)
Visible itchy rash	1.3; 2.1-5.3 (.7)	0.7; 0.2-2.4 (.6)	1.6; 0.3-8.2 (.6)
Baseline 1 vs 2	2.8; 0.7-11.5 (.2)	1.8; 0.5-6.5 (.4)	2.6; 0.5-11.6 (.2)
Model χ^2^ statistic for overall model fit	64.0 (.04)	34.2 (.005)	26.3 (.01)
AUC	0.66 (.01)	0.82 (.01)	0.84 (.01)

Controlling for “use of emollient before test reading,” “visible itchy rash at 2 months,” “infant sex,” and “infant birthweight.”
